# Onset of Spontaneous Ovarian Hyperstimulation Syndrome in the Third Trimester: Case Report

**DOI:** 10.7759/cureus.20940

**Published:** 2022-01-04

**Authors:** Rawan M Alqurashi, Shahad A Alsuwat, Maryam A Yamani, Salma Y Omar

**Affiliations:** 1 Medicine, Umm Al-Qura University, Makkah, SAU; 2 Obstetrics and Gynecology, Maternity and Children Hospital, Makkah, SAU

**Keywords:** ovarian cysts., polycystic ovarian syndrome, third trimester, ovulation induction, ovarian hyperstimulation syndrome

## Abstract

Ovarian hyperstimulation syndrome (OHSS) is a rare and occasionally fatal complication of ovulation induction. However, OHSS has occurred without interventional ovulation induction and in spontaneous ovulatory cycles. In most reported cases, physiological production of human chorionic gonadotropin was high, as in cases of multiple gestation, molar pregnancy, polycystic ovarian syndrome, and hypothyroidism. We report a very rare case of spontaneous OHSS in a healthy 36-year-old woman, gravida 5 para 2 + 2, 35 weeks pregnant, who had become pregnant naturally. According to our research, this is the first report of a case that occurred in the third trimester.

## Introduction

Ovarian hyperstimulation syndrome (OHSS) is a rare and occasionally fatal complication of ovulation induction (used in assisted reproductive technologies) in which the coexistence of multiple ovarian cysts with increased vascular hyperpermeability leads to a fluid shift from the intravascular to the extravascular space (third spacing), hypovolemia, and hemoconcentration [1,2]. It is classified as mild, moderate, severe, or critical depending on the signs, symptoms, laboratory test findings, and ultrasound findings [3].

Mild OHSS is characterized by bilateral ovarian enlargement and several follicular and corpus luteal cysts measuring up to 8 cm in diameter, as well as abdominal bloating and mild abdominal pain [3]. Moderate OHSS is marked by ovarian enlargement up to 12 cm, abdominal bloating due to ovarian enlargement, and gastrointestinal symptoms (e.g., nausea, vomiting, and diarrhea), as well as ultrasound evidence of ascites. The first indicator of moderate hyperstimulation could be a sudden weight gain of more than 3 kg [3]. Severe OHSS is defined by the presence of large ovarian cysts (> 12×12 cm), clinical ascites with or without hydrothorax, hyperkalemia (potassium > 5 mmol/L), hyponatremia (sodium < 135 mmol/L), hypo-osmolarity (osmolarity < 282 mOsm/kg), hypoproteinemia (serum albumin < 35 g/L), oliguria (< 300 mL/d or < 30 mL/h), creatinine 1.1 - 1.5 mg/dL, and hypovolemic shock. hemoconcentration with a hematocrit of more than 45 percent, a white cell count of more than 15000, liver dysfunction, increased blood viscosity, and thromboembolic events may occur [3].

Critical OHSS is marked by the presence of severe ascites or hydrothorax, hematocrit > 55%, white cell count > 25000/mL, oliguria or anuria, creatinine ≥ 1.6 mg/dL, creatinine clearance < 50 mL/min, thromboembolism, or acute respiratory distress syndrome [3]. On occasion, OHSS has occurred without interventional ovulation induction and during spontaneous ovulatory cycles; in most reported cases, physiological production of human chorionic gonadotropin was high, as in cases of multiple gestations, molar pregnancy, polycystic ovarian syndrome, and hypothyroidism [1]. The symptoms of spontaneous OHSS ordinarily occur between the eigth and 12th weeks of pregnancy, whereas in cases of iatrogenic OHSS, symptoms occur between the third and fifth weeks of pregnancy [2].

We report a very rare case of spontaneous OHSS that started during the third trimester in a woman who became pregnant naturally.

## Case presentation

A previously healthy 36-year-old woman, gravida 5 para 2 + 2, 35 weeks pregnant, was referred by a gynecology and obstetrics clinic to our hospital because a bilateral ovarian cyst was found incidentally on routine ultrasonography during the third trimester. The ultrasound findings were associated with bilateral abdominal discomfort and hirsutism, which had developed gradually during the third trimester. She had conceived spontaneously and denied having taken any ovulation-inducing agent, and the pregnancy was uneventful. During this pregnancy, the patient reported that during the first trimester, a small cyst in the right ovary was found incidentally on ultrasonography, and it resolved without intervention. In the third trimester, bilateral cysts appeared with enlargement of both ovaries (which were 5 cm in diameter); enlargement increased each week to 7, 11, and 12 cm.

Menarche had occurred at the age of 13 years. Two years before this pregnancy, her menstrual cycles became irregular, and the polycystic ovarian syndrome was diagnosed. It was managed with dydrogesterone due to secondary amenorrhea, and she had not taken contraception pills since that diagnosis, she had a history of two spontaneous abortions in the first trimester, which were managed conservatively, and two uncomplicated cesarean sections at term, the last one in 2017.

She was alert, oriented, well-nourished, and weighed 78 kg. Her temperature (36.5°C), pulse rate (109 bpm), and blood pressure (125/75 mmHg) were within normal limits. Pelvic examination revealed that the size of the uterus was compatible with the gestational age of the fetus, and large, mobile bilateral adnexal masses were found. Results of breast and thyroid examinations were normal. Pelvic ultrasonography revealed a single viable fetus, aged 35 weeks + 4 days with positive cardiac activity, and bilateral ovarian enlargement by multilocular cysts, most with clear content; the right ovary (Figure 1) measured 18.2 × 9.2 × 14.2 cm, and the left ovary (Figure 2) measured 14.85 × 10.67 × 11.5 cm. Some cysts on the left ovary were hemorrhagic, and no internal vascularity was observed in either ovary.

**Figure 1:** Right ovary Ultrasound scan of abnormally enlarged right ovary, depicting multiple cystic masses.

**Figure 2:** Left ovary Ultrasound scan of abnormally enlarged left ovary, depicting multiple cystic masses.

Laboratory studies revealed normal hemoglobin level (11.0 g/dL), mean corpuscular volume (77.7 fL), mean corpuscular hemoglobin level (24.3 pg), hematocrit level (35.1%), white blood cell count (6.93 × 103/mL), and platelet count (304 × 103/mL); normal levels of blood urea nitrogen (2.3 mmol/L), creatinine (52.3 mmol/L), random blood glucose (4.7 mmol/L), aspartate aminotransferase (14 U/L), alkaline phosphatase (216 U/L), total protein (65 g/L), and albumin level (31 g/L); and normal prothrombin time (12.70 s), partial thromboplastin time (26.5 s), and international normalized ratio (0.98). The patient's blood type was O Rhesus (Rh)-positive.

Spontaneous OHSS was diagnosed, prophylactic enoxaparin and paracetamol as needed were described. She was informed to be vigilant to these signs increasing abdominal distension or pain, shortness of breath, hypotension, palpitation, and decrease in urine output. The pregnancy continued without complications and without further signs of ascites. At 37 weeks and three days, the patient came to the emergency room with contracting lower abdominal pain. The cervix was dilated at 1 cm; an emergency cesarean section was performed, and a 3.600-kg baby girl was delivered with complete placenta and membranes. During surgery, large bilateral ovarian cysts were noted; the simple ovarian cysts were aspirated, and cystectomy was performed for the small right-sided hemorrhagic cysts. The ovarian size was then markedly reduced. Both fallopian tubes were normal. No complications occurred after the delivery, and at the two-months follow-up, the patient was doing well, with no new complaints.

## Discussion

The pathogenesis of OHSS is not fully understood. In most cases, it is an iatrogenic complication of ovulation induction therapy and infertility treatments such as clomiphene citrate (CC), human menopausal gonadotropin (hMG), purified follicle-stimulating hormone (FSH), and GnRH analogs (GnRH-a), manifesting as massive ovarian enlargement and the formation of multiple ovarian cysts [4]. However, spontaneous OHSS is extremely rare in natural pregnancies in the absence of such treatment [4].

Hyperstimulation of the enlarged ovaries causes excessive production of vasoactive substances, mainly vascular endothelial growth factor, which leads to an increase in vascular permeability and third spacing and results in intravascular hypovolemia with the concomitant development of lower limb edema; ascites; and, in severe cases, pleural effusion, diminished renal blood flow, and pericardial effusion [5]. Findings of numerous studies suggest that this syndrome occurs more frequently in cases of polycystic ovarian syndrome, hypothyroidism, twin pregnancy, and molar pregnancy [6,7]. Our patient had a history of polycystic ovarian syndrome but a singleton pregnancy.

Symptoms of spontaneous OHSS almost always occur between the eighth and 14th weeks of pregnancy, and those of iatrogenic OHSS appear earlier, between the third and fifth weeks [1]. To the best of our knowledge, this is the first report of a case that occurred in the third trimester.

OHSS is a self-limited disease. Management should be conservative and directed at symptoms. The main management options include thyroid hormone replacement for women with uncontrolled hypothyroidism, paracentesis for patients with significant ascites, thoracentesis for those with pleural effusion, and thromboembolism prophylaxis [7,8]. Data concerning later gestational complications in pregnancies complicated by OHSS are limited. Uncontrolled studies suggested that OHSS pregnancies had a higher rate of later complications, such as gestational diabetes and pregnancy-associated hypertension, and prematurity [9]. According to current studies, the pregnancy should be continued, and affected patients should be monitored closely [1].

## Conclusions

OHSS in most cases is a self-limited iatrogenic complication of ovarian stimulation; however, it may also happen spontaneously during pregnancy. Our case highlights the possibility of spontaneous OHSS in the third trimester, as well as the need of having a strong suspicion for OHSS when a clinical presentation is not explained by common medical conditions. The disease can be managed conservatively. In unusual cases, life-threatening complications may occur. To guarantee a positive outcome, early detection and adequate supportive care are recommended.
